# Clinical efficacy and mechanism of mesenchymal stromal cells in treatment of COVID-19

**DOI:** 10.1186/s13287-022-02743-0

**Published:** 2022-02-07

**Authors:** Kun Lu, Shi-tao Geng, Shikai Tang, Hua Yang, Wei Xiong, Fang Xu, Qijun Yuan, Xian Xiao, Renqiang Huang, Haihui Liang, Zhipeng Chen, Chuanyun Qian, Yang Li, Songqing Wang

**Affiliations:** 1 Department of Neurosurgery, First Naval Hospital of Southern Theater Command, Zhanjiang, 524000 China; 2 Department of Emergency, First Naval Hospital of Southern Theater Command, Zhanjiang, 524000 China; 3 Department of Emergency, First Affiliated Hospital of Kunming Medical University, Kunming, 650032 China

**Keywords:** Coronavirus disease 2019, Mesenchymal stromal cells, Clinical efficacy, Immunomodulation, Tissue repair

## Abstract

Coronavirus disease 2019 (COVID-19) is a highly infectious epidemic disease that has seriously affected human health worldwide. To date, however, there is still no definitive drug for the treatment of COVID-19. Cell-based therapies could represent a new breakthrough. Over the past several decades, mesenchymal stromal cells (MSCs) have proven to be ideal candidates for the treatment of many viral infectious diseases due to their immunomodulatory and tissue repair or regeneration promoting properties, and several relevant clinical trials for the treatment of COVID-19 have been registered internationally. Herein, we systematically summarize the clinical efficacy of MSCs in the treatment of COVID-19 based on published results, including mortality, time to symptom improvement, computed tomography (CT) imaging, cytokines, and safety, while elaborating on the possible mechanisms underpinning the effects of MSCs, to provide a reference for subsequent studies.

## Introduction

Coronavirus disease 2019 (COVID-19) is a highly infectious disease caused by severe acute respiratory syndrome coronavirus 2 (SARS*-*CoV*-*2). Based on available data, one of the hallmarks of SARS-CoV-2 infection pathogenesis is cytokine storm in the lung. Acute virus-induced cytokine release can lead to pulmonary edema, ventilatory dysfunction, and acute respiratory distress syndrome (ARDS) [1], especially in severe cases, which is characterized by the up-regulation of proinflammatory cytokines and chemokines, abnormal cellular immune response, respiratory and cardiovascular failure, end organ injury, and possibly death [2, 3]. To date, however, no specific antiviral drug has been proven effective in the treatment of COVID-19 and therefore is urgently required. A variety of strategies have been proposed to control cytokine storms and reduce mortality, such as selective cytokine blockade (e.g., anakinra or tocilizumab), JAK inhibition, intravenous immunoglobulin administration, mesenchymal stromal cell (MSC) therapy, and artificial blood purification [4, 5].

Based on the results of several models and stage-clinical trials of ARDS and sepsis, cell-based therapy, especially stem cell therapy, has emerged as a promising therapeutic area, especially for the treatment of COVID-19 [6–8]. MSCs are pluripotent cells obtained from different tissues, such as adipose and bone marrow. Due to their immunomodulatory properties, MSCs can alter immune cell function, modulate immune responses, and reduce inflammation-induced lung injury [9]. These cells can also prevent apoptosis and regenerate lung cells, especially type II alveolar cells, by producing growth factors such as keratinocyte growth factor (KGF), vascular endothelial growth factor (VEGF), and hepatocyte growth factor (HGF) [10]. Furthermore, by expressing indoleamine 2,3-dioxygenase (IDO), MSCs can stimulate interferon-γ (IFN-γ) production and IFN-γ-independent restriction of viral replication [11, 12]. Thus, the immunomodulatory, tissue repair, and antiviral properties of MSCs highlight their potential for the treatment of COVID-19 [10].

The safety and efficacy of MSCs have been demonstrated in multiple clinical trials related to the treatment of COVID-19 [6–8, 13]. As of October 2021, 51clinical trials for MSC-based COVID-19 therapy have been registered (http://clinicaltrials.gov/ and http://www.chictr.org.cn/) (Table 1). In this article, we summarize the findings of seven published clinical trials (Table 2) to help clarify the regulation of cytokines by MSCs in patients with COVID-19, and whether this therapy can improve patient symptoms, shorten hospital stays, and reduce mortality, in conjunction with a high safety and low adverse event profile. The underlying mechanisms by which MSCs may act are also explored, with the view to provide a reference for subsequent trials and research.

**Table 1:** Trial of registered MSCs in the treatment of COVID-19

Registration no	Title	Cell source	No. patients	Methods
ChiCTR2000029580	A prospective, single-blind, randomized controlled trial for Ruxolitinib combined with mesenchymal stem cell infusion in the treatment of patients with severe 2019-nCoV pneumonia	Ruxolitinib in combination with MSCs	35	NA
ChiCTR2000029990	Clinical trials of mesenchymal stem cells for the treatment of pneumonitis caused by novel coronavirus pneumonia (COVID-19)	MSCs	60	NA
ChiCTR2000030020	The clinical application and basic research related to mesenchymal stem cells to treat novel coronavirus pneumonia (COVID-19)	MSCs	20	NA
ChiCTR2000030088	Umbilical cord Wharton's Jelly derived mesenchymal stem cells in the treatment of severe novel coronavirus pneumonia (COVID-19)	Umbilical cord Wharton’s Jelly derived MSC	20	IV injection of Wharton's Jelly mesenchymal stem cells (1 × 10^6^/kg), cell suspension volume: 40 ml
ChiCTR2000030116	Safety and effectiveness of human umbilical cord mesenchymal stem cells in the treatment of acute respiratory distress syndrome of severe novel coronavirus pneumonia (COVID-19)	hUC-MSCs	16	Different stem cell doses (specific unknown)
ChiCTR2000030138	Clinical Trial for Human Mesenchymal Stem Cells in the Treatment of Severe Novel Coronavirus Pneumonia (COVID-19)	hUC-MSCs	30	NA
ChiCTR2000030173	Key techniques of umbilical cord mesenchymal stem cells for the treatment of novel coronavirus pneumonia (COVID-19) and clinical application demonstration	hUC-MSCs	30	NA
ChiCTR2000030261	A study for the key technology of mesenchymal stem cells exosomes atomization in the treatment of novel coronavirus pneumonia (COVID-19)	MSCs exosomes	13	Aerosol inhalation of exosomes(Specific unknown)
ChiCTR2000030484	HUMSCs and Exosomes Treating Patients with Lung Injury following Novel Coronavirus Pneumonia (COVID-19)	HU-MSCs and Exosomes	30	NA
ChiCTR2000030835	Clinical study for the efficacy of Mesenchymal stem cells (MSC) in the treatment of severe novel coronavirus pneumonia (COVID-19)	hUC-MSCs	20	NA
ChiCTR2000030866	Open-label, observational study of human umbilical cord-derived mesenchymal stem cells in the treatment of severe and critical patients with novel coronavirus pneumonia (COVID-19)	hUC-MSCs	20	Intravenous infusion of 1 × 10^6^ cells/kg/time on day 0, 3, 6
ChiCTR2000030944	Clinical study of human NK cells and MSCs transplantation for severe novel coronavirus pneumonia (COVID-19)	Human NK cells and MSCs transplantation	10	NA
ChiCTR2000031319	Safety and Efficacy Study of Allogeneic Human Dental Pulp Mesenchymal Stem Cells to Treat Severe novel coronavirus pneumonia (COVID-19) patients	Allogeneic Human Dental Pulp MSC	10	NA
ChiCTR2000031430	Clinical study of human umbilical cord mesenchymal stem cells in the treatment of novel coronavirus pneumonia (COVID-19)-induced pulmonary fibrosis	hUC-MSCs	100	4 × 10^7^/ times, intravenous injection on days 0, 3, and 6 for a total of 3 times
ChiCTR2000031494	Clinical study for stem cells in the treatment of severe novel coronavirus pneumonia (COVID-19)	MSCs	18	NA
NCT04252118	Safety and Efficiency of Mesenchymal Stem Cell in Treating Pneumonia Patients Infected With COVID-19	MSCs	20	3 times of MSCs(3.0 × 10^7^ MSCs intravenously at Day 0, Day 3, Day 6)
NCT04392778	What is the Effect of Mesenchymal Stem Cell Therapy on Seriously Ill Patients With Covid 19 in Intensive Care? (Prospective Double Controlled Study)	MSCs	30	3.0 × 10^6^ cells/kg (3 times, on Day 0, Day 3, Day 6)
NCT04269525	Clinical Research Regarding the Availability and Safety of UC-MSCs Treatment for Serious Pneumonia and Critical Pneumonia Caused by the 2019-nCOV Infection	UC-MSCs	16	3.3 × 10^7^ cell number / 50 ml / bag, 3 bags each time. on the 1st, 3rd, 5th, and 7th days after enrollment, 1 time each day
NCT04273646	Clinical Study of Human Umbilical Cord Mesenchymal Stem Cells in the Treatment of Severe COVID-19	UC-MSCs	48	4 times, 0.5 × 10^6^ cells/kg body weight intravenously at Day 1, Day 3, Day 5, Day 7
NCT04288102	A Phase II, Multicenter, Randomized, Double-blind, Placebo-controlled Trial to Evaluate the Efficacy and Safety of Human Umbilical Cord-derived Mesenchymal Stem Cells in the Treatment of Severe COVID-19 Patients	UC-MSCs	100	4.0 × 10^7^cells/times (3 times, Day 0, Day 3, Day 6.)
NCT04346368	Safety and Efficacy of Intravenous Infusion of Bone Marrow-Derived Mesenchymal Stem Cells in Severe Patients With Coronavirus Disease 2019 (COVID-19): A Phase 1/2 Randomized Controlled Trial	BM-MSCs	20	1 × 10^6^ /kg body weight intravenously at Day 1
NCT04397796	Phase 1b Randomized, Double-Blind, Placebo-Controlled Study Of The Safety Of Therapeutic Treatment With Immunomodulatory Mesenchymal Stem Cells In Adults With COVID-19 Infection Requiring Mechanical Ventilation	BM-Allo.MSC	45	NA
NCT04293692	Human Umbilical Cord Mesenchymal Stem Cells Treatment for Pneumonia Patients Infected by 2019 Novel Coronavirus	UC-MSCs	24	0.5 × 10^6^ cells/kg body weight suspended in 100 mL saline containing 1% human albumin intravenously at Day1, Day3, Day5, Day7
NCT04437823	Efficacy of Intravenous Infusions of Stem Cells in the Treatment of COVID-19 Patients	UC-MSCs	20	5 × 10^5^ cells/kg (3 times, Day 1, Day 3 and Day 5
NCT04456361	A Study of Mesenchymal Stem Cells as a Treatment in Patients With Acute Respiratory Distress Syndrome Caused by COVID-19	UC-MSCs	9	1 × 10^8^ cells/time (one time)
NCT04313322	Treatment of COVID-19 Patients Using Wharton's Jelly-Mesenchymal Stem Cells	WJ-MSCs	5	1 × 10^6^ cells/kg (3 times
NCT04390152	Safety and Efficacy of Intravenous Infusion of Wharton's Jelly Derived Mesenchymal Stem Cell Plus Standard Therapy for the Treatment of Patients With Acute Respiratory Distress Syndrome Diagnosis Due to COVID 19: A Randomized Controlled Trial	WJ-MSCs	40	50 × 10^6^ cells/time (2 times)
NCT04315987	Exploratory Clinical Study to Assess the Efficacy of NestaCell® Mesenchymal Stem Cell to Treat Patients With Severe COVID-19 Pneumonia	NestaCell® MSCs	90	A dose of 2 × 10^7^ cells will be administered IV on days 1, 3, 5 and 7
NCT04302519	Clinical Study of Novel Coronavirus-Induced Severe Pneumonia Treated by Dental Pulp Mesenchymal Stem Cells	Dental MSCs	24	1 × 10^6^ cells/kg (3 times, on Day1, Day 3 and Day 7)
NCT04276987	A Pilot Clinical Study on Aerosol Inhalation of the Exosomes Derived From Allogenic Adipose Mesenchymal Stem Cells in the Treatment of Severe Patients With Novel Coronavirus Pneumonia	MSCs-derived exosomes	24	5 times aerosol inhalation (2.0 × 10^8^ nanovesicles/3 ml at Day 1, Day 2, Day 3, Day 4, Day 5)
NCT04341610	Allogeneic Adipose Tissue-Derived Mesenchymal Stromal Cell Therapy for Treating Patients With Severe Respiratory COVID-19. A Danish, Double-blind, Randomized Placebo-controlled Study	A-MSCs	NA	100 million cells diluted in 100 ml saline
NCT04331613	Safety and Efficacy Study of Human Embryonic Stem Cells Derived M Cells (CAStem) for the Treatment of Severe COVID-19 Associated With or Without Acute Respiratory Distress Syndrome (ARDS)	CAStem	9	3 cohorts with 3 patients/cohort who receive doses of 3, 5 or 10 million cells/kg
NCT04339660	Clinical Research of Human Mesenchymal Stem Cells in the Treatment of COVID-19 Pneumonia	UC-MSCs	30	1 × 10^6^ cells /kg body weight suspended in 100 mL saline
NCT04336254	Safety and Efficacy Study of Allogeneic Human Dental Pulp Mesenchymal Stem Cells to Treat Severe Pneumonia of COVID-19: a Single-center, Prospective, Randomized Clinical Trial	Allogeneic Human Dental Pulp MSCs	20	Intravenous injection of 3.0 × 10^7^ human dental pulp stem cells solution (30 ml) on day 1, day 4 and day 7,
NCT04366323	Phase I / II Clinical Trial, Multicenter, Randomized and Controlled, to Assess the Safety and Efficacy of Intravenous Administration of Allogeneic Adult Mesenchymal Stem Cells of Expanded Adipose Tissue in Patients With Severe Pneumonia Due to COVID-19	Adipose tissue-derived mesenchymal stem cells	26	8 × 10^7^ cells/time (two times)
NCT04349631	Phase II, Open Label, Single-Center, Clinical Trial to Assess Efficacy of HB-adMSCs to Provide Immune Support Against Coronavirus Disease	HB-adMSCs	56	Five times (dose not applicable)
NCT04366063	Mesenchymal Stem Cell Therapy for Acute Respiratory Distress Syndrome in Coronavirus Infection: A Phase 2–3 Clinical Trial	MSCs	60	1 × 10^8^ cells with or without extracellular vesicles (EVs) in two times (on Day 0, Day 2 for MSC and on Day 4, Day 6 for EVs)
NCT04352803	IV Infusion of Autologous Adipose-Derived Mesenchymal Cells for Abatement of Respiratory Compromise in SARS-CoV-2 Pandemic (COVID-19)	Autologous adipose MSC's (AMSCs)	20	500,000/kg IV
NCT04362189	A Randomized, Placebo-Controlled, Double-Blind, Efficacy and Safety Study of Allogeneic HB-adMSCs for the Treatment of COVID-19	HB-adMSC	100	100 million cells/dose(4 times, day 0, 3, 7, and 10)
NCT04348461	Two-treatment, Randomized, Controlled, Multicenter Clinical Trial to Assess the Safety and Efficacy of Intravenous Administration of Expanded Allogeneic Adipose Tissue Adult Mesenchymal Stromal Cells in Critically Ill Patients COVID-19	Allogeneic and expanded adipose-derived MSCs (AMSCs)	100	1.5 × 10^6^ cells/kg (two times)
NCT03042143	Repair of Acute Respiratory Distress Syndrome by Stromal Cell Administration (REALIST): An Open Label Dose Escalation Phase 1 Trial Followed by a Randomized, Double-blind, Placebo-controlled Phase 2 Trial (COVID-19)	Human umbilical cord-derived CD362-enriched MSCs	120	Maximum tolerated dose from the phase 1 trial will be infused over 30 to 90 min
NCT04361942	Double-Blind, Placebo-controlled, Phase II Trial to Evaluate Safety and Efficacy of Allogenic Mesenchymal Stromal Cells MSV_allo for Treatment of Acute Respiratory Failure in Patients With COVID-19 Pneumonia (COVID_MSV)	MSCs	24	Intravenous injection of 1 million MSV cells/Kg diluted in 100 ml saline
NCT04333368	Cell Therapy Using Umbilical Cord-derived Mesenchymal Stromal Cells in SARS-CoV-2-related ARDS	UCMSCs	47	1 × 10^6^ cells/kg (three times, Day 1, Day 3 and Day 5)
NCT04416139	Mesenchymal Stem Cells for the Treatment of Severe Acute Respiratory Distress Syndrome Due to COVID-19. Pilot Study	MSCs	10	1 million cells/Kg in a single dose
NCT04428801	Clinical Study for the Prophylactic Efficacy of Autologous Adipose Tissue-Derived Mesenchymal Stem Cells (AdMSCs) Against Coronavirus 2019 (COVID-19)	autologous adipose-derived stem cells	200	Three doses of 200 million cells via intravenously infusion every three days
NCT04348435	A Randomized, Double-Blind, Single Center, Efficacy and Safety Study of Allogeneic HB-adMSCs to Provide Immune Support Against COVID-19	Allogeneic HB-adMSCs	55	200 × 10^6^ cells/time (5 times, Day 0, Day 2, Day 6, Day 10 and Day 14)
NCT04444271	Prospective, Randomized Phase 2 Clinical Trial of Mesenchymal Stem Cells(MSCs) for the Treatment of Coronavirus Disease 2019(COVID-19)	MSCs	20	2 × 10^6^ cells/kg (two times, Day 1 and Day7
NCT04429763	Safety and Efficacy of Mesenchymal Stem Cells in the Management of Severe COVID-19	UCBMSCs	30	One dose of 1 × 10^6^ cells/Kg
NCT04490486	Phase I, Randomized, Double-Blinded, Placebo Control Study to Evaluate the Safety and Potential Efficacy of Intravenous Infusion of Umbilical Cord Tissue (UC) Derived Mesenchymal Stem Cells (MSCs) Versus Placebo to Treat Acute Pulmonary Inflammation Due to COVID-19 With Moderate to Severe Symptoms	UCMSCs	21	100 × 10^6^ cells/time (two times, Day 1 and Day 3)
NCT04457609	Application of Umbilical Cord Mesenchymal Stem Cells as Adjuvant Therapy for Critically-Ill COVID-19 Patients	UCMSCs	40	1 × 10^6^ cells/kgBW in 100 cc of 0.9% NaCl for 1 h
NCT04486001	COVID-19 Stem Cell Therapy: A Phase I Study of Intravenous Administration of Allogeneic Adipose Stem Cells	PSC-04	20	NA

**Table 2:** Summary of published clinical trials of MSCs in the treatment of COVID-19

Registration No	Country		Patients		Types of trials		Age(control/MSC)		Sex (M/F)		Number(control/MSC)			Methods
ChiCTR2000031494	China		Severe		A single-center open-label, individually randomized, standard treatment-controlled trial		57.86 ± 15.79/61.00 ± 17.87		24/19		29/12			Intravenous administration was used. Before the intravenous drip, the hUC-MSCs were suspended in 100 ml of normal saline, and the total number of transplanted cells was calculated as 2 × 106 cells/kg. The infusion was from the patients’ right cubital veins and lasted approximately 1 h (35 drops/min)
NA	Iran		ARDS		A phase 1, two-center, open-label, single-arm trial		53.80 ± 10.37		8/3		11			The UC-MSCs were suspended in 100 ml normal saline with 5% w/w human serum albumin for each infusion. The PL-MSCs were suspended in 100 ml of normal saline supplemented with 2% w/w human serum albumin for each infusion. Three intravenous infusions (200 × 10^6^ cells) every other day for a total of 600 × 10^6^ cells. (UC-MSCs; 6 cases) or (PL-MSCs; 5 cases). The infusion time was approximately 30–45 min at a speed of approximately 50 drops/min
NCT04252118	China		Moderate, severe		A parallel assigned controlled, non-randomized, phase 1 clinical trial				11/7		9/9			Received three cycles of intravenous infusion of allogeneic UC-MSCs (3 × 10^7^cells each infusion) on days 0, 3, and 6. The total volume of the UC-MSCs infusion was 60 ml
NCT04288102		China		Severe		A randomized, double-blind, placebo-controlled phase 2 trial		59.94/60.72		56/44		35/65	The treatment dose was 4.0 × 10^7^ cells for each procedure, and three procedures were carried out for each patient on day 0, 3, and 6 after randomization. Infusion was started with a standard blood filter tubing set with a pore size of 170 μm. Under electrocardiographic monitoring, the cell product was infused by gravity within 60 min	
NCT04392778		Turkey		Critical ill		A prospective double-controlled trial				19/11		10/10/10	Three consecutive doses on treatment days 0, 3, and 6, (as 3 × 10^6^cells/kg, intravenously)	
ChiCTR2000029606		China		Severe, critically ill		A multicenter, open-label, nonrandomized, and parallel controlled phase I clinical trial		61.11/58.31		30/14		18/26	Menstrual blood-derived MSC were administered as three infusions totaling 9 × 10^7^MSCs every other day (day 1, day 3, and day 5). Each infusion contained 3 × 107cells resuspended in 500 mL saline solution and was performed at a speed of 30–40 drops/min for about 15 min, followed by a speed of 100–120 drops/min for 2 h to retain MSC vitality	
NCT04355728		USA		ARDS		A double-blind, phase 1/2a, randomized controlled trial		58.83 ± 11.61/58.58 ± 15.93		13/11		12/12	Two intravenous infusions of 100 ± 20 × 10^6^UC-MSCs each, in 50 mL vehicle solution containing human serum albumin and heparin, infused over 10 ± 5 min, at days 0 and 3	

## Efficacy

### Mortality

According to the World Health Organization (WHO), the cumulative number of deaths due to COVID-19 has surpassed 5.5 million globally. Multiple studies have shown that MSC therapy can significantly reduce the incidence and mortality of critical illness (Table 3) [14–19]. For example, Shu et al. [14] found the mortality in the MSC treatment group was zero. In addition, Xu et al. [17] reported significantly higher survival in patients treated with MSC (92.31%) than those in the routine treatment group (66.67%). Another study reported a 28-day survival rate of 91% in MSC-treated patients compared with 42% in non-treated controls, with the control group also showing a higher risk of death (hazard ratio (HR) 8.76; 95% CI 1.07–71.4) [18]. Furthermore, serious adverse event-free survival showed significant improvement with MSC treatment compared with the controls (HR 6.22; 95% CI 1.33–28.96). Thus, the above results confirm the safety of MSC therapy and its effectiveness at reducing mortality and improving survival. However, due to the small sample sizes in the above studies, data from large-scale clinical phase 3 trials are still required.

**Table 3:** Clinical efficacy of MSCs in the treatment of COVID-19

Authors	Mortality (control/MSC)	Systemic changes and symptoms	CT Imaging	Inflammatory cytokines
Shu et al	28-day mortality rate was 10.34% / 0	Clinical symptoms obviously improved beginning on the third day of stem cell infusion. The time to clinical improvement in the hUC-MSC treatment group was shorter than that in the control group (median, 9.0 days vs. 14.0 days)	CT scores, the number of lobes involved, GGO, and consolidation were significantly better than those in the control group	IL-6 and CRP rapidly reduced Lymphocyte count return to normal levels in less time
Hashemian et al	Five cases died 4–19 days (average: 8 days) after the first cell infusion	The clinical symptoms of most surviving patients improved significantly	In the surviving cases, the shadow area on lung CT was significantly reduced	Pro-inflammatory decreased including IL-8, TNF-α, CRP, IL-6, INF-ɣ Anti-inflammatory cytokines including IL-4 and IL-10 levels increased
Meng et al	All 18 patients recovered and were discharged from hospital	In most severe patients, the PaO2/FiO2 ratio improved	The lung lesions were well controlled within 6 days, and completely faded away within 2 weeks after UC-MSCs transfusion	There was a reduced trend in the levels of all these cytokines within 14 days (IFN-γ, TNF-α, MCP-1, IP-10, IL-22, IL-1RA, IL-18, IL-8 and MIP-1)
Shi et al	NA	6-min walking distance was longer in the MSC group (median 420.00 m) than in the placebo group (median 403.00 m) oxygen therapy maximum forced VCmax and DLCO, the six-category scale, status of oxygen therapy, and mMRC dyspnea score were similar between the two groups	Total lesion proportion (%) of the whole lung volume as measured by CT were decreased	No significant difference in the subsets of peripheral lymphocyte counts (CD4 + T cells, CD8 + T cells, B cells, NK cells) and plasma markers between the two groups
Adas et al	Mortality rate was 60%/30%	NA	NA	Serum ferritin, fibrinogen and CRP levels had significantly decreased IL-6, IFN-γ, IL-2, IL-12, and IL-17A significant decrease No statistically significant decrease in IL-β and TNF-α levels IL-10, IL-13, and IL-1ra levels significant increase MMP-9 and MMP-3 levels were decreased Growth factors TGF-β, VEGF, KGF, and NGF levels were increased
Xu et al	Mortality rate was 33.33%/7.69%	Average improvement time (8.80 ± 10.77 vs 3.00 ± 3.05. No significant differences in length of stay or ICU days. No significant difference in the incidence of shock or multiple organ failure	One month after MSC infusion, 85.00% patients in the experimental group had improved,50.00% patients in the control group had improved	NA
Lanzoni et al	Survival was improved in the UC-MSC vs the control group: 91% vs 42%. SAE-free survival was significantly improved in the UC-MSC group	Time to recovery was significantly shorter in the UC-MSC treatment group	NA	GM-CSF, IFN-γ, IL-5, IL-6, IL-7, TNF-α, TNF-β, PDGF-BB, and RANTES were statistically significant decreases from day 0 to day 6 only in the UC-MSC treatment group

### Systemic changes and symptoms

MSC treatment can significantly shorten the time to clinical symptom improvement in COVID-19 patients. Lanzoni et al. [18] showed a significantly shorter COVID-19 recovery time following MSC treatment, with an HR for recovery of 0.29 (95% CI 0.09–0.95) in the control group versus the MSC-treated group. Several other studies have also demonstrated that MSC therapy can significantly expedite patient recovery. A recent experiment comparing pulmonary function recovery and comprehensive reserve capacity based on a 6-min walk test (6-MWT) found that walk distance was longer in MSC-treated patients compared with the controls, although maximal forced vital capacity (VCmax), diffusing lung capacity for carbon monoxide (DLCO), six category scale, oxygen therapy status, and mMRC dyspnea score did not differ significantly between the two groups [20]. In critically ill patients, the partial pressure of arterial oxygen: percentage of inspired oxygen (PaO_2_/FiO_2_) ratio showed improvement after MSC treatment [16]. Furthermore, MSC-treated patients demonstrated significant improvement in clinical symptoms and were discharged from the ICU within 2–7 days after MSC infusion, with significant relief of dyspnea, decrease in respiratory rate within 48–96 h, and improvement in oxygen saturation [15]. Shu et al. [14] also reported significant improvements in weakness, fatigue, shortness of breath, and low oxygen saturation in MSC-treated patients compared with the controls.

In addition to clinical symptoms, laboratory parameters have also been examined [15, 16], including C-reactive protein (CRP), alanine aminotransferase (ALT), creatinine, serum ferritin (SF), and platelet levels, which all returned to their normal range after MSC administration. These results suggest that MSCs not only improve pulmonary symptoms but also positively impact the functional recovery of multiple organs, such as the liver and kidney.

### Computed tomography (CT) imaging

As clinical symptoms are influenced by multiple factors, and the evaluation of symptom relief is subjective, various researchers have assessed lung lesions in COVID-19 patients using imaging. Studies using CT imaging have reported that time of pulmonary lesions is significantly shortened in patients treated with MSCs. A single-center, open-label, randomized, standard treatment-controlled trial showed that CT score, number of lobes affected, ground glass opacity, and solid changes were significantly improved in MSC-treated patients compared with the controls [14]. In another study, the rate of chest imaging changes 1 month after MSC infusion was significantly improved in 85% of MSC-treated patients compared to 50% of control-group patients [17]. Previous research also reported that lung lesions were well controlled within 6 days and completely disappeared within 2 weeks after MSC infusion [16]. A phase 2 clinical trial also reported a significant decrease in total lesion proportion in the whole lung measured by CT from baseline to day 28 after MSC infusion [20].

### Cytokines

Cytokine storms are considered one of the main characteristics of COVID-19. To date, however, no definitive therapy has been shown to completely control cytokine storm or restore organ damage caused by infection with SARS*-*CoV*-*2. MSC transplantation may act as an immunomodulator in the development of cytokine storm caused by inflammation. Therefore, many scholars believe that MSCs have a decided advantage in controlling cytokine storm induced by COVID-19.

Several published clinical trials indicate that MSCs can effectively control the expression of inflammatory cytokines in COVID-19 patients [14–16, 18, 19]. Several studies have reported that proinflammatory cytokines, such as interleukin (IL)-8, tumor necrosis factor (TNF)-α, CRP, IL-6, INF-γ, IL-2, IL-12, and IL-17A, decreased significantly after MSC infusion, while anti-inflammatory cytokines IL-4 and IL-10 increased significantly [14, 15, 18]. However, other research reported that IL-β and TNF-α levels were not significantly reduced after MSC administration [19]. In addition, a clinical trial reported no significant changes in cytokines, but a reduced trend in cytokine levels within 14 days (IFN-γ, TNF-α, monocyte chemokine-1 (MCP-1), interferon inducible protein-10 (IP-10), IL-22, IL-1RA, IL-18, IL-8, and MIP-1) [16]. Intragroup analysis found that granulocyte macrophage colony stimulating factor (GM-CSF), IFN-γ, IL-5, IL-6, IL-7, TNF-α, TNF-β, platelet derived growth factor-BB (PDGF-BB), and RANTES decreased significantly from days 0 to 6 in the UC-MSC treatment group [18]. These data, to some extent, demonstrate the effect of MSC treatment in patients with COVID-19, and the differences in outcomes between trials may be due to differences in disease degree and age. Thus, the results of large-scale phase 3 trials should help further define the role of MSCs in treatment.

### Safety

Drug and treatment safety must be considered in clinical application. Recently, the clinical outcome of a 65-year-old female patient with COVID-19 treated with allogeneic human umbilical cord blood-derived MSCs (UCB-MSCs) was reported, with no adverse events noted during treatment and was well tolerated [21]. Hashemian et al*.* also reported that the liver and kidney function of patients were not affected during MSC infusion [15]. Another study found that MSCs can cure or significantly improve the functional results of patients without obvious adverse events [22]. These results illustrate, to some extent, the safety of MSCs for the treatment of COVID-19, but the number of included experimenters is small and lack of randomized controlled trials. In view of this, many clinical trials have begun to evaluate the safety, feasibility, and tolerability of MSCs.

Various trials suggest that MSC therapy is safe for COVID-19. A prospective double-controlled trial reported no adverse or serious adverse events related to MSC treatment [19]. Another phase 1 clinical trial evaluated the safety of MSC infusion in patients with moderate to severe COVID-19 and reported that three patients experienced adverse effects, although these events were considered to be caused by disease progression based on pre-existing symptoms [16]. Similarly, two clinical randomized controlled trials [18, 20] showed that the overall incidence of adverse events was similar in the MSC and control groups, but these events were largely unrelated to treatment, and significantly more subjects experienced serious adverse events in the control group than in the MSC group. Thus, the above findings reflect the safety of MSC therapy and its potential benefits at reducing COVID-19-related adverse events.

In general, although the safety of MSCs is acceptable, treatment may not be applicable to some COVID-19 patients with serious complications. For example, a phase 1 trial [15] showed that multiple infusions of high-dose allogeneic MSCs were safe and rapidly improved respiratory distress and reduced inflammatory biomarkers in some cases of critically ill COVID-19-induced ARDS, but four patients with multiple organ failure or sepsis died within 5–19 days (mean 10 days) after the first MSC infusion. These findings suggest that contraindications need to be strictly considered when selecting patients for MSC therapy.

### Mechanisms of COVID-19 treatment with MSCs

Several studies [23–27] have shown that MSCs can be safely infused intravenously or via the endobronchial route in humans, thus allowing MSCs to accumulate in the lungs to improve the lung microenvironment, protect alveolar epithelial cells, protect against pulmonary fibrosis, and improve lung function [28–30]. Although the specific molecular mechanisms underlying the effects of MSCs on COVID-19 treatment require further research, several studies have investigated possible processes, as summarized below.

### Immunomodulation

MSCs exhibit strong immunomodulatory potential. Their immunomodulatory functions are mainly exerted through cell-to-cell contact, paracrine secretion, endocrine action, and immune cell interactions (e.g., T cells, B cells, natural killer (NK) cells, macrophages, monocytes, dendritic cells (DCs), and neutrophils). Thus, MSCs participate in both innate and adaptive immunity [31–33], with regulatory T cell (Treg) and monocyte interactions appearing to play a key role [34]. Of course, it may vary according to the pathological mechanism of the disease, source of MSCs, and route of administration.

MSCs show immunosuppressive effects when exposed to sufficiently high levels of pro-inflammatory cytokines [35], but can promote an inflammatory response under low levels of TNF-α and IFN-γ [35]. Thus, MSCs may need to be triggered by inflammatory cytokines to become immunosuppressive, and the inflammatory environment may be a key factor affecting immunoregulation of MSCs. One of the characteristics of COVID-19 is the formation of an inflammatory cytokine storm, which may provide an inflammatory environment for the immunomodulation of MSCs.

After infusion of MSCs in COVID-19 patients, IL-1RA, IL-6, HGF, prostaglandin E2 (PGE2) secreted by MSCs promoted monocyte/macrophage differentiation into anti-inflammatory/immunomodulatory (type 2) phenotype, and directly inhibited differentiation into type 1 phenotype and DCs [36, 37]. On the one hand, type 2 monocytes/macrophages secrete high levels of IL-10, reduce expression levels of IL-12p70, TNF-α, and IL-17, prevent monocytes from differentiating into DCs, and convert monocytes into an anti-inflammatory, IL-10-secreting subtype via a positive feedback loop [36], while high levels of IL-10 inhibit T cell activity [38]. On the other hand, macrophages release more CCL-18 and transforming growth factor-β1 (TGF-β1) during differentiation into type 2 macrophages, which helps induce Treg formation, while CCL-18 converts memory CD4^+^T cells into CD4^+^CD25^+^Foxp3^+^Treg cells and increases IL-10 and TGF-β1 generation [39–41]. Furthermore, it was observed in the asthma model that the infused MSCs was engulfed by pulmonary macrophages, resulting in a shift of monocytes to a type 2 immunosuppressive phenotype, polarization of CD14^++^CD16^−^ classical monocytes to a CD14^++^CD16^+^CD206^+^ immunoregulatory intermediate subset with anti-inflammatory properties, and increased expression of IL-10 and programmed death ligand-1 (PD-L1) [42–44], thereby driving the immune response toward an anti-inflammatory response.

MSCs act on the adaptive immune system, particularly T cells [32, 33], in various ways, e.g., inhibition of the proliferation, cytokine secretion, and cytotoxicity of T cells and regulation of T helper 1 (Th1)/T helper 2 (Th2) balance and Treg function. MSCs can induce IL-10 and PGE2 production and inhibit IL-17, IL-22, and IFN-γ levels to limit Th17 differentiation [45] and suppress Th17 responses by modulating the IL-25/STAT3/PD-L1 axis [46]. Upon interaction with DCs, MSCs can cause a shift from pro-inflammatory Th1 cells to anti-inflammatory Th2 cells [47]. Induction of CD4^+^CD25^+^Foxp3^+^ Tregs is one of the main features of MSC-mediated immune regulation, and MSCs can secrete TGF-β1 and IDO to induce the formation of Tregs [39, 47]. MSCs can directly interact with B cells and promote the generation of regulatory B cells (Bregs), which secrete IL-10 to convert effector CD4^+^T cells into Foxp3^+^Tregs [48, 49]. MSCs can also exert direct immunosuppressive effects on T cell behavior by suppressing CD4^+^T cell activation via the secretion of PD-L, including PD-L1 and PD-L2 [50, 51].

### Promotion of tissue repair and regeneration

In addition to their immunomodulatory properties, the multilineage differentiation ability of MSCs also makes them ideal candidates for cell therapy. Numerous studies have demonstrated the regenerative capacity of MSCs in musculoskeletal system, nervous system, cardiac muscle, liver, cornea, trachea, and skin tissue repair [52].

COVID-19 is characterized by lung tissue damage, which can cause systemic multi organ damage, especially in patients who develop ARDS. After injection, MSCs can differentiate into lung tissue or secrete factors (e.g., angiopoietin-1 (ANGPT1), EGF, VEGF, PGE2, HGF, VEGFA, KGF, and IL-10) that can induce host repair/regenerative mechanisms [53], promote epithelial and endothelial repair, increase alveolar fluid clearance, regulate lung epithelial and endothelial permeability, and reduce inflammation in patients with ARDS lung injury [52, 54, 55]. In addition, these factors can promote tissue repair by supporting the growth and differentiation of local stem/progenitor cells, regulating the deposition of extracellular matrix molecules, stimulating anti-scarring pathways, and inducing neovascularization [56, 57]. Induction factors secreted by MSCs, such as VEGF, brain-derived neurotrophic factor (BDNF), and TGF-β1, can promote the development of self-repair. Activin A, EGF, KGF, HGF, and IGF-2 play important roles in MSC differentiation into epithelial cells by triggering appropriate signaling pathways [58, 59]. MSCs also show anti-apoptotic effects [53], and the release of KGF and HGF by MSCs can protect alveolar epithelial cells from apoptosis by increasing B-cell lymphoma-2 (BCL-2) expression and inhibiting hypoxia-inducible factor-1α (HIF-1α) protein expression [60]. Furthermore, the expression of various factors, such as VEGF, HGF, and TGF-β, can reverse endothelial cell apoptosis [61].

The immunomodulatory properties and tissue repair/regeneration abilities of MSCs highlight their potential in the treatment of COVID-19. MSCs can also exert antibacterial effects by secreting soluble mediators to reduce the number of bacteria, improve the antibacterial response of immune cells, and inhibit the migration of proinflammatory cells into infected tissues [53]. Thus, MSCs can participate in the inhibition of viral replication via different mechanisms [11, 12].

## Conclusions

As cells with multilineage differentiation ability, MSCs are potential candidates for cell-based therapy to treat COVID-19. Various clinical trials have demonstrated the efficacy and safety of MSCs for the treatment of COVID-19 patients, especially critically ill patients, not only improving clinical symptoms, hospital stay, cytokine release, and mortality, but also showing a high safety profile with limited adverse events. However, further evidence from large-scale and long-term phase 3 clinical trials is still required. Although the therapeutic action of MSCs in COVID-19 patients appears to involve immunomodulation, promotion of repair/regeneration, and inhibition of viral replication through cell-to-cell contact and paracrine activity, the specific mechanism needs further investigation. However, we expect more data from currently progressing trials should support the role of MSCs in COVID-19.

## Data Availability

Not applicable.

## Abbreviations

COVID-19: Coronavirus disease 2019
MSCs: Mesenchymal stromal cells
*SARS-CoV-2*: Severe acute respiratory syndrome coronavirus *2*
ARDS: Acute respiratory distress syndrome
KGF: Keratinocyte growth factor
VEGF: Vascular endothelial growth factor
HGF: Hepatocyte growth factor
IDO: 2,3-Dioxygenase
IFN: Interferon
AE: Adverse event
6-MWT: 6-Minute walk test
VCmax: Maximal forced vital capacity
DLCO: Diffusing lung capacity for carbon monoxide
PaO2/FiO2: Pressure of arterial oxygen: percentage of inspired oxygen
CRP: C-reactive protein
ALT: Alanine aminotransferase
SF: Serum ferritin
*GGO*: Ground glass opacity
IL: Interleukin
TNF: Tumor necrosis factor
MCP-1: Monocyte chemokine-1
IP-10: Interferon-inducible protein-10
GM-CSF: Granulocyte macrophage colony stimulating factor
PDGF-BB: Platelet-derived growth factor-BB
NK: Natural killer
DCs: Dendritic cells
PGE2: Prostaglandin E2
TGF-β1: Transforming growth factor-β1
PD-L1: Programmed death ligand-1
ANGPT1: Angiopoietin-1
EGF: Epidermal growth factor
BDNF: Brain-derived neurotrophic factor
BCL-2: B-cell lymphoma-2
HIF-1α: Hypoxia-inducible factor-1α
